# Adaptive Neuro-Fuzzy Determination of the Effect of Experimental Parameters on Vehicle Agent Speed Relative to Vehicle Intruder

This article has been retracted.

**DOI:** 10.1371/journal.pone.0155697

**Published:** 2016-05-24

**Authors:** Shahaboddin Shamshirband, Lejla Banjanovic-Mehmedovic, Ivan Bosankic, Suad Kasapovic, Ainuddin Wahid Bin Abdul Wahab

**Affiliations:** 1 Department of Computer System and Information Technology, Faculty of Computer Science and Information Technology, University of Malaya, Kuala Lumpur, Malaysia; 2 Department of Automation and Robotics, Faculty of Electrical Engineering, University of Tuzla, Tuzla, Bosnia and Herzegovina; 3 Department of Telecommunication, Faculty of Electrical Engineering, University of Tuzla, Tuzla, Bosnia and Herzegovina; Southwest University, CHINA

## Abstract

Intelligent Transportation Systems rely on understanding, predicting and affecting the interactions between vehicles. The goal of this paper is to choose a small subset from the larger set so that the resulting regression model is simple, yet have good predictive ability for Vehicle agent speed relative to Vehicle intruder. The method of ANFIS (adaptive neuro fuzzy inference system) was applied to the data resulting from these measurements. The ANFIS process for *variable selection* was implemented in order to detect the predominant variables affecting the prediction of agent speed relative to intruder. This process includes several ways to discover a subset of the total set of recorded parameters, showing good predictive capability. The ANFIS network was used to perform a variable search. Then, it was used to determine how 9 parameters (Intruder Front sensors active (boolean), Intruder Rear sensors active (boolean), Agent Front sensors active (boolean), Agent Rear sensors active (boolean), RSSI signal intensity/strength (integer), Elapsed time (in seconds), Distance between Agent and Intruder (m), Angle of Agent relative to Intruder (angle between vehicles °), Altitude difference between Agent and Intruder (m)) influence prediction of agent speed relative to intruder. The results indicated that distance between Vehicle agent and Vehicle intruder (m) and angle of Vehicle agent relative to Vehicle Intruder (angle between vehicles °) is the most influential parameters to Vehicle agent speed relative to Vehicle intruder.

## Introduction

Cyber-Physical Systems (CPS) is emerging as an integrative research field aimed toward a new generation of engineered systems [1]. CPSs are mostly distributed parameter systems (DPSs) which combine real-time computing, embedded systems, wireless sensor networks, control theory, signal processing and knowledge creation using artificial intelligence [2].

Intelligent Transport systems (ITS) fall in the framework of cyber-physical systems due to the interaction between physical systems (vehicles) and a distributed information gathering and dissemination infrastructure. Electrical and hybrid vehicles are recognized as an important ingredient in a high-efficiency and clean transportation network. The Energy Storage System (ESS) largely affects the performance and cost of an electric vehicle, especcially if the vehicles are treated as a component of the Cyber-physical systems, where the energy saving is important.

Intelligent Transportation Systems rely on understanding, predicting and affecting the interactions between vehicles. Development of such systems must be based upon data derived from actual wireless vehicle-to-vehicle (V2V) and vehicle-to-infrastructure (V2I) communications in real world applications. There are many applications in ITS which are being developed based upon vehicle to vehicle and vehicle to infrastructure communication [3]: vehicle tracking, collision avoidance, controller design and cooperative driving challenges. Understanding of how these interactions affect, for example on speed profile of vehicles, flow or travel time is also necessary to create robust systems. Speed profile can be estimated from historical data through analyzing limited traffic information from fields. For instance, the traffic data, such as distance, location, etc. from vehicle (agent) could be linked with historical travel speed data.

The cooperative intelligent transport system (C-ITS) have recently received a lot of attention. A cooperative behaviour includes two or more actors working towards a common or mutually beneficial goal, purpose, or benefit; enabled by interaction and information exchange between the actors [4]. Cooperative behaviour involves actions such as exchange of system state information, interaction about intentions, planned behaviours, etc. Typical goals within the transport system context are, the improvement of safety and increased transport efficiency.

In [5], a set of vehicles is connected via wireless communication with the infrastructure to exchange information related to the road segment along which the vehicle is traveling, the goal being to increase road safety. Within C-ITS, information is shared between many actors such as vehicles, infrastructures, cloud services, etc. However, only sharing information is not enough to be considered a C-ITS, cooperation and interaction between the actors in the system is also required [4].

Accurate prediction of traffic information is important in many applications in Intelligent Transport systems in order to reduce the uncertainty of the future traffic states, improve traffic mobility, providing the driver with a realistic estimation of travel times and expected delays, and alternative routes to the destinations or to improve. There are many research in traffic information predictions such as speed, flow and travel time [6–10]. In order to fulfill the driving performance requirements and ensuring operational safety in an electric vehicle, energy storage estimation model is of great significance for battery electric vehicles [11–13].

Variable or feature selection have become the focus of much research in areas of application for which datasets with tens or hundreds of thousands of variables are available. The *variable selection*, includes a number of ways to discover a subset of the total recorded parameters that show good capability of prediction. The objectives of variable selection are: improving the prediction performance of the predictors, providing faster and more cost-effective predictors and providing a better understanding of the underlying process that generated the data [14]. A more advanced approach considered the variable selection problem using artificial neural networks [15–18], ANFIS [19], genetic algorithms [20–21], a principal component analysis [22]or experimentally investigated through the well-adopted Electrochemical Impedance Spectroscopy (EIS) technique [23].

This paper focus on constructing and selecting subsets of features that are useful to build a good speed predictor in Intelligent Transport systems. The Adaptive neuro-fuzzy Inference Technique (ANFIS) was applied to the resulting data to select the most influential parameters affecting the Vehicle agent speed relative to Vehicle intruder prediction. The ANFIS network was used to perform a variable search and thereafter, it was used to examine how9 parameters (Intruder Front sensors active (boolean), Intruder Rear sensors active (boolean), Agent Front sensors active (boolean), Agent Rear sensors active (boolean), RSSI signal intensity/strength (integer), Elapsed time (in seconds), Distance between Agent and Intruder (m), Angle of Agent relative to Intruder (angle between vehicles °), Altitude difference between Agent and Intruder (m)) influence prediction of agent speed relative to intruder.

The rest of this paper is organized as follows. Section II describes the used methodology. In Section III results of ANFIS based variables selection for Vehicle agent speed relative to Vehicle intruder prediction are presented to demonstrate the effectiveness of the proposed approach. Finally, Section IV gives the main concluding remarks of the paper.

## Methodology

### Variable selection techniques

To build a system with the best characteristics, it is necessary to identify the most relevant and influential subset of parameters and subject these to analysis. This process of selection is usually called variable selection. In a typical prediction task, there may be a large number of candidate variables available that could be used for building an automatic predictor [24]. If this number of candidate variables is denoted with *n*, the variable selection problem is defined as selecting *d < n* variables (the optimal subset of variables), that allow the construction of the best predictor. There can be many reasons for selecting only a subset of the variables: it is cheaper to measure only d variables; prediction accuracy might be improved through exclusion of irrelevant variables; the predictor to be built is usually simpler and potentially faster when less input variables are used; knowing which variables are relevant can give insight into the nature of the prediction problem.

Many heuristic algorithms have been proposed for the variable selection problem. Sequential Search (SS) is a meta-heuristic method aimed at finding optimal subsets of variables for a specified model size [25]. The basic idea is to replace each variable at a time with all the remaining ones and see whether a better model is obtained. An alternative approach to the variable selection problem is via the utilization of a genetic algorithm (GAs) [26]. The method is a general one that can be applied in a wide variety of domains [21]. Differently from GA, Particle Swarm Optimization (PSO) method don't compete but cooperate in order to find the optimal solution. PSO was initially thought as an optimization method and was only later modified in order to be specifically applied to variable selection [27].

One of the most important issues in using neural networks for the analysis of real-world problems is the input variable selection problem [28]. Neural networks are an architecture which is made up of extremely parallel adaptive processing elements. These are interconnected through structured networks. Therefore, the accuracy of the neural network models which are created as a result of this data rely heavily on the accuracy of the chosen sensor data in the representation of the system. Artificial Neural network (ANN)has been extensively used to model complex nonlinear dynamic systems, which can be emulated by feeding a measured database into the configured network to train the ANN neurons until either an acceptable precision or the maximum iteration number is reached. Although an ANN is often trained using limited experimental data, it possesses an inherent ability to identify and respond to patterns that are not the same as the ones with which it was trained. A well-trained ANN can be resilient to highly uncertain and even noise-perturbed input data while still generating accurate outputs. To achieve a successful generation and creation of a model which is capable to estimate a special process output, the selection process of the subset of parameters that are really pertinent is crucial. This is achieved in the process of variable selection.

Amongst the many neural network system, one of the most used and powerful is the ANFIS; and the ANFIS was employed here, for the purposes of this study, in the variable selection part [29]. ANFIS, a hybrid intelligent system that increases the capability of learning and adapting automatically has been used by researchers for many different purposes [30–35]. There are many advantages in the use of the ANFIS scheme. Some of the main advantages are: it is adaptable to optimization and adaptive methods, as well as being computationally efficient. ANFIS can be integrated with professional systems and rough sets for use in other applications. And here is yet another favorable aspect of ANFIS, it conducts the tedious job of training membership functions.

In order to determine how the a few main parameters affect the vehicle agent speed relative to vehicle intruder, a parameter search by employing the ANFIS was conducted.

### Variable selection using ANFIS

Generating predetermined input-output subsets requires the construction of a set of fuzzy ‘IF THEN’ rules with the suitable MFs(membership function). The ANFIS can serve as the foundation for such a construction. The input-output data are converted membership functions. In accordance to the collection of input-output data, the ANFIS takes the initial FIS and adjusts it through a back propagation algorithm. The FIS is comprised of three components, (1) a rule base, (2) a database and (3) a reasoning mechanism. The rule base consists of a choice of fuzzy rules. The database assigns the MFs which are employed in the fuzzy rules. Finally, the last component is the reasoning mechanism and it infers from the rules and input data to come to a feasible outcome. These intelligent systems are a combination of knowledge, methods and techniques from a variety of different sources. They adjust to perform better in environments which are changing. These systems have similar-human intelligence within a specific domain. The ANFIS recognizes patterns and assists in the revision of environments. FIS integrates human comprehension, does interfacing, and makes decisions.

FIS in MATLAB is employed in the whole process of the FIS training and evaluation. An ANFIS network for 2 input variables is the most influential parameters on the vehicle agent speed relative to vehicle intruder prediction. This is depicted in Fig 1.

**Fig 1:** ANFIS structure.

The fuzzy IF-THEN rules of Takagi and Sugeno’s class and two inputs for the first-order Sugeno is employed for the purposes of this study:

$$if\;x\;is\;A\;and\;y\;is\;C\;then\;f_{1}=p_{1}x+q_{1}y+r_{1}$$ (1)

The 1stlayer is made up of input parameters MFs, and it provides the input values to the following layer. Each node here is considered an adaptive node having a node function *O = μ*_*AB*_(*x*) and *O = μ*_*CD*_(*x*) where *μ*_*AB*_(*x*) and *μ*_*CD*_(*x*) are membership functions. Bell-shaped membership functions having themaximum value (1.0) and the minimum value (0.0) areselected, such as,

$$\mu \left(x\right)=bell\left(x;a_{i},b_{i},c_{i},d_{i}\right)=\frac{1}{1+{\left[{\left(\frac{x-c_{i}}{a_{i}}\right)}^{2}\right]}^{b_{i}}}$$ (2)

where {*a*_*i*_, *b*_*i*_, *c*_*i*_, *d*_*i*_} is the set of parameters set. The parameters of this layer are designated as premise parameters. Here, *x* and *y* are the inputs to nodes. They represent a combined version of the two most impactful variableson the vehicle agent speed relative to vehicle intruder prediction.

The membership layer is the second layer. It looks for the weights of every membership function. This layer gets the receiving signals from the preceding layer and then it acts as membership function to the representation of the fuzzy sets of each input variable, respectively. Second layer nodes are non-adaptive.The layer acts as a multiplier for the receiving signals and sends out the oucomein *w*_*i*_ = *μ*_*AB*_(*x*) * *μ*_*CD*_(*y*) form. Every output nodeexhibits the firing strength of a rule.

The next layer, the third, is known as the rule layer. All neurons here act as the pre-condition matching the fuzzy rules. Each rule’s activation level is calculated whereby the number of fuzzy rules is equal to the quantity of layers. Every node computes the normalized weights. The nodes in the 3rd layer are also considered non-adaptive.each of the node computes the value ofthe rule’s firing strength over thesum of all rules’ firing strengths in the form of $w_{i}^{*}=\frac{w_{i}}{w_{1}+w_{2}}$, *i* = 1, 2. The outcomes are refered to as the normalized firing strengths.

The 4^th^layer is responsible for providing the output values as a result of the inference of rules. This layer is also known as the defuzzification layer. Every 4th layer node is an adaptive node having the node function $O_{i}^{4}=w_{i}^{*}xf=w_{i}^{*}\left(p_{i}x+q_{i}y+r_{i}\right)$. In this layer, the {*p*_*i*_, *q*_*i*_, *r*} is the variable set. The variable setis designated as the consequent parameters.

The 5th and final layer is known as the output layer. It adds up all the receiving inputs from the preceding layer. Thereafter, it converts the fuzzy classification outcomes into a binary (crisp). The single node of the5th layer is considered non-adaptive. This node calculates the total output as the wholesum of all receiving signals,

$$O_{i}^{5}=\sum_{i}w_{i}^{*}xf=\frac{{\sum^{\text{​}}}_{i}w_{i}f}{{\sum^{\text{​}}}_{i}w_{i}}$$ (3)

In the process of identification of variables in the ANFIS architectures, the hybrid learning algorithms were applied. The functional signals progress until the 4^th^ layer whereby the hybrid learning algorithm passes. Further, the consequent variables are found by the least squares estimation. In the backward pass, the error rates circulate backwards and the premise variables are sychornized through the gradient decline order.

## Experimental Work

### Data collection

We used data from a detailed Warrigal dataset, presented in paper [3]. This rich dataset, derived from the interactions of large trucks and smaller 4WD vehicles in an industrial setting, and was collected by a fleet of 13 vehicles operating in a large quarry-type environment during a period of 3 years. The data span a period of 3 years with a resolution of 1 hertz. Due to its size, the dataset is divided into daily periods. Peer-to-peer communication between vehicles is effected on two frequencies to improve redundancy through the complementary properties of each frequency. All vehicles communicate on 2.4 GHz and 433 MHz. Light vehicles are fitted with a single 2.4 GHz antenna and a single 433 MHz antenna. Heavy vehicles are fitted with a single 2.4 GHz antenna at the front of the vehicle and a pair of 433 MHz antennas, one mounted at the front and the other at the rear.

Warrigal dataset contains vehicle state information, vehicle-to-vehicle communications and road maps at high temporal resolution for large numbers of interacting vehicles over a long time. Analyzing of interactions number between agent-intruder pairs, we selected 4 pairs from top list (Vehicle agent, Vehicle Intruder: (48, 74); (48,47); (48,52) and (48,42), Table 1) and make dataset with 300–400 samples for each pair in both directions.

**Table 1:** Number of interactions between different vehicles pairs (agent, intruder).

Vehicle agent ID	Vehicle intruder ID	Number of interactions
48	74	65301
74	48	61745
48	47	38590
47	48	35824
48	52	37834
52	48	37375
48	42	37177
42	48	33569
…	…	…
75	50	10451
47	51	2990
48	75	111

### Input and output variables

Selected input and output parameters for variable selection analysis are presented on Fig 2.

**Fig 2:** Selected input and output parameters for analysis.

Table 2 shows the 9 input parameters selected for analysis(Intruder Front sensors active (boolean), Intruder Rear sensors active (boolean), Agent Front sensors active (boolean), Agent Rear sensors active (boolean), RSSI signal intensity/strength (integer), Elapsed time (in seconds), Distance between Agent and Intruder (m), Angle of Agent relative to Intruder (angle between vehicles °), Altitude difference between Agent and Intruder (m)). These parameters are considered potentially influential on agent speed relative to intruder in Table 3.

**Table 2:** Input parameters.

Input	Parameters description
1	Intruder Front sensors active (boolean)
2	Intruder Front sensors active (boolean)
3	Agent Front sensors active (boolean)
4	Agent Rear sensors active (boolean)
5	RSSI signal intensity/strength (integer)
6	Elapsed time (in seconds)
7	Distance between Agent and Intruder (m)
8	Angle of Agent relative to Intruder (angle between vehicles °)
9	Altitude difference between Agent and Intruder (m)

**Table 3:** Output parameters.

Output	Parameters description
1	Vehicle agent speed relative to Vehicle intruder

## Results and Discussion

As mentioned before, the purpose of this procedure is to find a subset of the total set of parameters that have been recorded to show good capability of prediction. The problems faced in the process of the selection of parameters could possibly be resolved by integrating and applying prior knowledge to segregate and remove parameters that are irrelevant. The objective here is to select the proper explanatory (input) parameters and thereby reduce and minimize the error that exists between the observed values and the model estimations of the explained variables.

A comprehensive search was performed from the given inputs in order to choose the set of the ultimate optimal combination inputs, Table 2 which has the most impact and influence on the output parameter (vehicle agent speed relative to vehicle intruder prediction), Table 3. Basically, an ANFIS model is built by the functions for each combination and they are then respectively trained for single epoch. Subsequently, the achieved performance is reported. From the outset, the most impactful input in the prediction of the output was identified and determined, as depicted in Table 4. The input variables with the smaller training error have the most relevance in regards to the outcome.

**Table 4:** Every input parameter’s influence on vehicle agent speed relative to vehicle intruder prediction.

Influences of selected input parameters on output prediction	Influences of selected input parameters on output prediction
1^st^sample	2^nd^sample
ANFIS model 7: in7 -->trn = 2.5132, chk = 2.6776	ANFIS model 7: in7 -->trn = 1.6329, chk = 3.7887
3^rd^sample	4^th^sample
ANFIS model 7: in7 -->trn = 2.1854, chk = 2.3523	ANFIS model 7: in7 -->trn = 1.9938, chk = 2.1650
5^th^sample	6^th^sample
ANFIS model 8: in8 -->trn = 2.7524, chk = 2.7489	ANFIS model 8: in8 -->trn = 1.9759, chk = 2.1625
7^th^sample	8^th^ sample
ANFIS model 8: in8 -->trn = 2.5803, chk = 3.0961	ANFIS model 8: in8 -->trn = 1.9926, chk = 2.4791

As it can be clearly seen from the results depicted in Table 4, the input variables 7 and 8 is the most influential for the vehicle agent speed relative to vehicle intruder prediction. The fact that both the checking errors and training are comparable is an indirect indication that suggests that there is no over fitting. This means that the selection of more than one input parameter in the construction of the ANFIS model can be explored. For the verification purposes, a look at the best integration of 2 receiving parameters can be conducted. The results listed in Table 5 show the optimal combinations of two input attributes for the prediction of the vehicle agent speed relative to vehicle intruder. Two optimal two inputs parameters can be then extracted for further analyzing.

**Table 5:** Combinations of two input parameters for vehicleagent speed relative to vehicle intruder prediction.

Influences of selected combinations of input parameters on output prediction	Influences of selected combinations of input parameters on output prediction
1^st^sample	2^nd^sample
ANFIS model 34: in7 in8 -->trn = 2.1454, chk = 2.6909	ANFIS model 31: in6 in7 -->trn = 1.3513, chk = 136.6236
3^rd^sample	4^th^sample
ANFIS model 34: in7 in8 -->trn = 1.7905, chk = 9.9407	ANFIS model 28: in5 in7 -->trn = 1.6388, chk = 2.7641
5^th^sample	6^th^ sample
ANFIS model 34: in7 in8 -->trn = 2.2627, chk = 3.3060	ANFIS model 34: in7 in8 -->trn = 1.6528, chk = 5.4500
7^th^sample	8^th^sample
ANFIS model 34: in7 in8 -->trn = 2.2725, chk = 2.8984	ANFIS model 34: in7 in8 -->trn = 1.8243, chk = 2.3537

To enable the ANFIS to find the right inputs quickly, the used function for all variables only trains each one for a single epoch. Once the inputs are fixed, the 100 epochs that are the quantity of epoch on ANFIS training can then be increased. Further, error curves for these 100 epochs of training and checking for two extracted input parameters.

The graph of the model for the ANFIS input-output (decision) surface for prediction of the vehicle agent speed relative to vehicle intruder prediction is a monotonic non-linear surface as shown in Fig 3. The figure below also shows the response of ANFIS model for the varying selected input parameters 7 and 8.

**Fig 3:** ANFIS decision surfaces for vehicle agent speed relative to vehicle intruder prediction for two selected parameters 7 (Distance between vehicles) and 8 (Relative Angle between vehicles).

## Conclusion

The recent developments in variable selection have addressed the problem of improving the performance of predictors. They have met the challenge of operating on input spaces of several thousand variables. There can be drawbacks in the inclusion of many input variables. Some of the drawbacks would include the difficulty in explaining the model, distractions and inaccuracies caused by irrelevant parameters, which consequently deteriorates the generalization capacity of the model, thus making data collecting more time-costly. However, methods that permit the reduction of the number of input variables can be figured out. If they reduce the model complexity, they are very useful. They incorporate better predictions and insights in the relevance of the variables.

The task of training an ANN and GA becomes more difficult in the case of real-world applications. Using varibale selection with ANFIS, with hybrid learning method, the training algorithm may determine a near-global optimum error, which decreases to the computational burden of model development.

The study carried out a systematic approach to select the most dominant parameters to predict the vehicle agent speed relative to vehicle intruder by the ANFIS methodology. The ANFIS network was used to determine how 9 parameters (Intruder Front sensors active (boolean), Intruder Rear sensors active (boolean), Agent Front sensors active (boolean), Agent Rear sensors active (boolean), RSSI signal intensity/strength (integer), Elapsed time (in seconds), Distance between Agent and Intruder (m), Angle of Agent relative to Intruder (angle between vehicles °), Altitude difference between Agent and Intruder (m)) influence prediction of agent speed relative to intruder. The results indicated that distance between Agent and Intruder (m) and angle of agent relative to Intruder (angle between vehicles °) is the most influential parameters to agent speed relative to intruder. The simulations also employed MATLAB, and outcomes were checked on the corresponding output blocks.

## Supporting Information

S1 File Supporting Information file rssi4874X. (XLSX)

S2 File Supporting Information file rssi5248X. (XLSX)

S3 File Supporting Information file rssi7448X. (XLSX)

S4 File Supporting Information file rssi4248X. (XLSX)

S5 File Supporting Information file rssi4748X. (XLSX)

S6 File Supporting Information file rssi4842X. (XLSX)

S7 File Supporting Information file rssi4847X. (XLSX)

S8 File Supporting Information file rssi4852X. (XLSX)

S1 Table Number of interactions between different vehicles pairs (agent, intruder). (DOCX)

S2 Table Input parameters. (DOCX)

S3 Table Output parameters. (DOCX)

S4 Table Every input parameter’s influence on vehicle agent speed relative to vehicle intruder prediction. (DOCX)

S5 Table Combinations of two input parameters for vehicleagent speed relative to vehicle intruder prediction. (DOCX)
